The article "Influence of Melatonin Treatment on Emotion, Sleep, and Life Quality in Perimenopausal Women: A Clinical Study" was retracted in 2023. Reasons: signs of a paper mill; compromised peer review; unreliable results or conclusions.

# Influence of Melatonin Treatment on Emotion, Sleep, and Life Quality in Perimenopausal Women: A Clinical Study

**DOI:** 10.1155/2023/2198804

**Published:** 2023-10-10

**Authors:** Jianfu Zhang, Bengui Jiang

**Affiliations:** ^1^Department of Pharmacy, Ningbo Women and Children's Hospital, Ningbo 315012, China; ^2^Department of Gynecology, Ningbo Women and Children's Hospital, Ningbo 315012, China

## Abstract

**Method:**

100 healthy perimenopausal women were recruited and randomly assigned to two groups, with 50 subjects in each group. In the control group, placebo was administrated daily for 3 cycles (4 weeks of treatment for 1 cycle and drug withdrawals for 1 week). The study group received 3 mg oral melatonin treatment daily in the same period of time. All subjects completed the study. We compared the uterine volume, endometrial thickness, LH (luteinizing hormone), FSH (follicle generating hormone), E2 (estradiol), and melatonin levels during daytime between the two groups before and after the study. Moreover, perimenopause syndrome, sleep, mood, and QoL were analyzed at the baseline and 3 cycles by the questionnaires of the Kupperman index, the Pittsburgh sleep quality index (PSQI), the Hamilton anxiety scale (HAMA), and the Hamilton depression scale (HAMD), as well as menopausal QoL (MENQOL), respectively. Any adverse reactions experienced by the subjects were also compared in the study. Finally, 91 participants (92%) completed the whole study, 47 and 44 in the study and control groups, respectively, and their data were considered in subsequent analyses.

**Results:**

After therapy, the two groups were similar in the uterine volume and endometrial thickness. In contrast to the control group, the study group showed notably decreased LH and FSH levels. No notable difference was discovered in E2 and melatonin levels between the two groups in the study. Moreover, the study group exhibited a significantly lower score in the Kupperman index, PSQI, HAMA, HAMD, and MENQOL scale than the control group. Moreover, the two groups had no notable difference in adverse reactions.

**Conclusion:**

Melatonin was a useful treatment to relieve climacteric symptoms and improve sleep, mood, and life quality in perimenopausal women without obvious adverse reactions.

## 1. Introduction

Perimenopause is defined as the period of time before and after menopause. It is suggested that the onset of menopause is associated with the ovarian failure and decreased estrogen, leading to hypothalamic-pituitary-ovarian (HPO) dysfunction and central nervous system involvement [1]. Due to fluctuations and deficiencies in reproductive hormones (estrogen and progestogen), women at this stage may be vulnerable to suffer from a series of symptoms, including physical (e.g., hot flushes, palpitations, and tachycardia) and psychological symptoms, such as anxiety, depression, sleep disorder, and cognitive decline [2]. The changing of reproductive hormones was thought to be responsible for the symptoms, and related therapy was the most widely used treatment for over 50 years. However, while hormone therapy has been proved to be effective in improving the symptoms, it remains controversial. A growing number of studies focusing on long-term outcomes suggested that hormone therapy is not suitable for all women, and it may increase the risk of cardiovascular events or breast cancer in those who are already at risk [3–5]. Thus, many new treatments have been developed in recent years.

Melatonin, primarily synthesized in the pineal gland, is an endogenous hormone, and its synthesis and secretion follow a circadian rhythm, which is inhibited during the day and stimulated at night [6]. Its concentration decreases with age, especially during the perimenopausal period [7]. In addition, melatonin has a close relationship with reproductive hormones, and it may exert an inhibitory effect through the HPO axis [8]. For instance, an animal experiment reported reduced plasma LH and 17-beta-estradiol after 60 days of melatonin administration in rats, and sex steroid receptors in the oviduct, ovary, as well as uterus were regulated differently [9]. Maganhin et al. [10] observed a correlation between melatonin and ovarian function, suggesting that it might take a crucial part in the production of reproductive hormone. Thus, it is plausible to speculate that melatonin is involved in menopause transition. Previous studies demonstrated that melatonin treatment can effectively improve the thyroid function and gonadotropin level and relieve menopause-related sleep and mood symptoms in perimenopausal or menopausal women [11–14]. However, a recent meta-analysis found that melatonin could improve physical symptoms, but it had little effect on general menopausal symptoms, estradiol levels, body mass index, sleep, and mood symptoms in menopausal women [15]. Early intervention with administration of melatonin in perimenopausal women seems to be more effective in alleviating the symptoms and may modify the transition of menopause in women.

Therefore, this study aimed at probing into the impacts of 3 mg melatonin daily in perimenopausal women. We speculated that melatonin treatment could help perimenopausal women relieve climacteric symptoms, mood, and sleep disorders and further improve their quality of life (QoL).

## 2. Methods

### 2.1. Participants

100 healthy perimenopausal women were enrolled originally from the outpatient department of the Ningbo Women and Children Hospital. All participants were 45–55 years Chinese women. They should experience (1) climacteric symptoms, including hot flashes, sleep disorder, anxiety, and depression, for less than 1 year and (2) irregular menstruation and have at least one menstruation in the past 6 months. The participants would be excluded if they conformed to one of these criteria: diagnosis of cardiovascular endocrine and gynecological diseases (hypertension, diabetes, gynecological malignancies, breast tumors, and other diseases), major somatic disease, substance abuse, current use or discontinuation of health care drugs, or reproductive hormone treatment for less than one month. Then, all participants were grouped into study and control groups in a random way (each *n* = 50) by a random number table. The study was performed with the permission of the Ethics Committee of the Ningbo Women and Children Hospital (No. S009, 2018), and informed consent was signed by each participant.

### 2.2. Clinical Assessment

Climacteric symptoms were scored with the Kupperman index, a 3-points scale with 11 items in their sequence of importance. Scores ranged from 15–19, 20–34, >34 indicating the degree of severity of the symptoms as mild, moderate, and severe, respectively [16]. The severity of depressive and anxiety symptoms were assessed through the Hamilton depression scale (HAMD, total score with a range of 0–75) [17] and the Hamilton anxiety scale (HAMA, total score with a range of 0–56) [18]. The Pittsburgh sleep quality index (PSQI) was adopted for evaluating overall sleep quality with a total score between 0 and 21. Besides, current QoL was evaluated by the menopausal quality of life (MENQOL), which contains 32 climacteric symptoms across 4 areas, including vasomotor, physical, sexual, and psychosocial symptoms [19]. The abovementioned questionnaires were provided for all participants before and after treatment.

### 2.3. Collection and Usage of Serum Samples

Blood samples were acquired from all fasting women through venous puncture on the day of completion of the questionnaires at the baseline and after treatment during daytime to allow the samples to stand for at least 30 minutes (indoor temperature). Then, the blood was treated by centrifugation to separate serum that was then kept at −20°C until use. The concentrations of melatonin, LH, FSH, and E2 level were analyzed by radioimmunoassay with kits manufactured by Immuno Biological Laboratories (Hamburg, Germany).

### 2.4. Intervention

Subjects randomly assigned to the study group (*n* = 50) were administered for 3 cycles (4 weeks of treatment for 1 cycle and drug withdrawals for 1 week) melatonin (3 mg in the evening) [20]. Subjects in the control group (*n* = 50) were given oral placebo (in the evening) in the same period of time. Placebo and melatonin were made into identical capsules, using lactose only or melatonin. All subjects were advised to take capsules before bedtime. When dispensing melatonin/placebo, the researchers were aware of the group.

### 2.5. Statistical Analysis

SPSS 25.0 (IBM Corp, Armonk, NY) was adopted for statistical processing. Intergroup comparisons of demographic and clinical data at the baseline were conducted via the independent sample *t*-test or chi-squared test, with *p* < 0.05 regarded as significant. For post-treatment data, an independent sample *t*-test and paired *t*-test were performed for intergroup and intragroup comparisons, respectively. The threshold was set as *p* < 0.05.

## 3. Results

### 3.1. Participants' Characteristics

Demographic characteristics were summarized in Table 1. The two groups presented no notable difference in the duration of perimenopausal state (*p*=0.90), age (*p*=0.87), BMI (*p*=0.53), history of alcohol (*p*=0.74), or smoking (*p*=0.71).

### 3.2. Uterine Volume and Endometrial Thickness

The two groups showed no notable differences in uterine volume at the baseline (*p*=0.74) and after treatment (*p*=0.76) and also showed no difference in endometrial thickness at the baseline (*p*=0.40) and after treatment (*p*=0.90). Moreover, the intragroup analysis showed no notable difference in uterine volume (*p*=0.23) and endometrial thickness (*p*=0.34) before and after treatment in the treatment group nor in the control one (uterine volume: *p*=0.89 and endometrial thickness: *p*=0.79). The details are shown in Table 2 and Figure 1.

### 3.3. Hormone Level

No notable difference was found between the two groups in LH, FSH, E2, and melatonin levels at the baseline. After treatment, the study group showed significantly decreased LH (*p* < 0.01) and FSH levels (*p* < 0.01) in contrast to the control group. In addition, notably decreased LH (*p* < 0.01) and FSH levels (*p* < 0.01) were found in the study group after treatment. The results are summarized in Table 3 and Figure 2.

### 3.4. Kupperman and MENQOL Scores

As shown in Figure 3 and Table 4, no notable difference was found in Kupperman and MENQOL scores between the two groups at the baseline. After treatment, the study group exhibited significant decreased scores in Kupperman (*p* < 0.01) and MENQOL (*p* < 0.01) scales in contrast to the control group. Furthermore, both groups showed significant reductions in Kupperman (study group: *p* < 0.01, control group: *p* < 0.01) and MENQOL scores (study group: *p* < 0.01, control group: *p* < 0.01) after treatment in contrast to those at the baseline.

### 3.5. HAMD, HAMA, and PSQI Scores

The two groups were similar in HAMD, HAMA, and PSQI scores at the baseline. After treatment, the study group showed significantly decreased scores in HAMD, HAMA, and PSQI scales in contrast to the other. Moreover, the study group exhibited significant decrease in HAMD (*p* < 0.01), HAMA (*p* < 0.01), and PSQI scores (*p* < 0.01) after treatment in contrast to those at the baseline. The details are shown in Table 5 and Figure 4.

### 3.6. Adverse Reactions

The two groups presented no notable differences with regard to the incidence of adverse reactions, including breast pain, rash, nausea, and vomiting (Table 6).

## 4. Discussion

An age-related decline in melatonin concentration was observed in aging healthy people, which might be bound up with pineal aging [21]. Prior research has revealed that melatonin treatment has a positive effect on climacteric symptoms, sleep, and mood disorder in perimenopausal and postmenopausal women and can circumvent the limitations of hormone therapy to some extent [22–24]. In this study, a 12-week melatonin administration in 100 perimenopausal women was conducted, with the main purpose of exploring its effect on sleep disorders, mood, and QoL. Our findings suggested that melatonin improved the abovementioned symptoms associated with perimenopausal and may have a regulatory effect on reproductive hormones without obvious adverse reactions.

As menopause approaches, women's ovarian function gradually degrades, resulting in a decreased sensitivity to gonadotropin and decreased estrogen levels [25]. Imbalance of hormone levels causes dysfunction of the autonomic nervous system, leading to a series of climacteric symptoms, such as heart palpitations, night sweats, and hot flashes, accompanied by mood and sleep disturbances. Perimenopause is the critical period for women to transition to menopause. Follow-up studies reported that women mood disorders (depression and anxiety) were more likely to occur during the menopausal transition than during the premenopausal phase. A higher risk of mood disorders may be related to the increased FSH and LH levels, as well as increased estradiol and FSH variability [26–28]. In this study, we found a notable decrease in FSH and LH in perimenopausal women treated with melatonin, which was consistent with previous findings. Converging evidence indicated that melatonin may be involved in the regulation of reproductive hormones by HPO axis and act directly on reproductive organs, such as reducing oxidative damage to follicles and promoting ovulation [29], as well as regulates the ovarian function through a receptor-mediated pathway [30]. Together with our results, these findings suggested that melatonin may be able to stabilize reproductive hormone imbalance to a certain extent during the perimenopausal period and play a role in relieving climacteric symptoms. However, the two groups in the study presented no notable difference in the E2 level. We speculated that it might be related to the intervention duration and dosage of melatonin treatment. Another plausible reason was individual differences in hormone secretion. Further long-term interventions at different doses in a larger sample size are required for confirming our hypothesis. After treatment, the two groups showed no notable difference in the serum melatonin concentrations, which may indicate that the use of melatonin does not increase the serum melatonin concentration during daytime and would not lead to adverse reactions. In addition, melatonin was considered to have an inhibitory effect on tumors. Regelson and Pierpaoli [31] revealed that melatonin may be involved in preventing the growth of tumors, especially hormone-sensitive ones. This inhibitory effect on cancer cells may depend on its antioxidant, immune stimulation, and apoptosis properties [32]. We observed no notable difference in uterine volume and endometrial thickness between the control and study groups after therapy. This may suggest that melatonin use does not elevate the risk of endometrial disease and breast cancer. However, whether melatonin has a protective effect on the reproductive organs and prevents the occurrence and development of tumors still needs further research.

The Kupperman index and MENQOL scores may reflect the severity of climacteric symptoms and their impact on life in the perimenopausal and menopausal women. Significant lower scores in these two scales were observed in the study group than in the control group after melatonin treatment in the study. Besides, we also observed a notable decrease in the two scale scores in both groups before and after treatment. These may indicate that melatonin use can effectively relieve climacteric symptoms and improve their QoL in the perimenopausal women, and placebo may have positive implications for the participants as well. As mentioned before, ovarian aging and the fluctuation and imbalance of reproductive hormone levels are responsible for the dysfunction of the autonomic nervous system and further cause the occurrence of climacteric symptoms. In this study, we found that melatonin may have a stabilizing effect on the imbalance of reproductive hormones without adverse reaction, which may be the main reason for the improvement of climacteric symptoms. Obviously, it makes sense that the women in the study group experienced an improvement in their QoL as their symptoms diminished.

Sleep disturbances is common during menopausal transition and postmenopausal state [33–35]. Previous studies suggested that women often report dissatisfaction with sleep quality, which may be related to vasomotor symptoms rather than age. As menopause progresses, women are more likely to experience sleep-onset insomnia or sleep-maintenance insomnia [36, 37]. Brown and Gervais [38] utilized a translational approach to investigate the contribution of ovarian hormones to sleep. They pointed that E2 loss may reduce its inhibitory effect on the cerebral cortex, leading to sleep disturbances. Moreover, it is well known that melatonin, a neurohormone that regulates the circadian rhythm of the sleep-wake cycle, decreases with age, which can cause sleep problems [39, 40]. Although no notable change was observed in the E2 level in the study group after treatment, the findings supported that melatonin can directly improve nighttime sleep. The improvement in physical symptoms and sleep would alleviate mood disorder and then would further enhance the QoL for perimenopausal women. A randomized control study reported that melatonin may have a positive effect on depression in perimenopausal and postmenopausal women [41]. A recent study confirmed the effect of melatonin on mood disorder, sleep, and QoL, as well as preventing bone loss [42]. HAMD and HAMA are clinically used to evaluate depression and anxiety, respectively. Similar to prior research, in the study, we found notably lower HAMD and HAMA scores in the study group than in the other group. Though changes in melatonin have been speculated to be associated with a series of mood symptoms, especially postpartum depressive symptoms [43, 44], the role of melatonin in psychiatric disorders such as major depressive disorder should be examined carefully considering its integrative specificities across metabolism, immunity, neurotransmission, and more. However, pharmacologic doses of melatonin can indeed result in significant impacts on both cognitive and motor performances and mood, in addition to the sleepiness it caused [45]. Despite the short range of action, melatonin has the potential to be directly affecting mood and emotion on its own. Therefore, our results provide new evidence that melatonin can relieve sleep and mood disorders and improve QoL.

The primary limitations of the study include a comparatively small sample size and certain heterogeneity of the sample. In addition, we did not measure nocturnal melatonin concentrations in the study to explore the effect of exogenous melatonin on reproductive hormones at night. Even so, we suggested that melatonin may be a suitable treatment for relieving climacteric symptoms while also improving sleep disorders, mood, and QoL in perimenopausal women. Our findings are promising for improving the symptoms in perimenopausal women and need to be confirmed in larger longitudinal studies.

## Figures and Tables

**Figure 1:** Uterine volume and endometrial thickness in the two groups before and after therapy. (a) Uterine volume in the study and control groups before and after therapy. (b) Endometrial thickness in the study and control groups before and after therapy.

**Figure 2:** LH, FSH, E2, and melatonin level before and after treatment in the two groups. LH: luteinizing hormone, FSH: follicle generating hormone, and E2: estradiol. (a) LH level in the study and control groups before and after therapy. (b) FSH level in the study and control groups before and after therapy. (c) E2 level in the study and control groups before and after therapy. (d) Melatonin level in the study and control groups before and after therapy. ^*∗∗*^*p* < 0.01.

**Figure 3:** Kupperman and MENQOLscores in the two groups before and after therapy. MENQOL: the menopausal quality of life (a). Kupperman scores in the study and control groups before and after therapy. (b). MENQOL scores in the study and control groups before and after therapy. ^*∗∗*^*p* < 0.01.

**Figure 4:** HAMD, HAMA, and PSQI scores in the two groups before and after treatment. HAMD: the Hamilton depression scale, HAMA: the Hamilton anxiety scale, and PSQI: the Pittsburgh sleep quality index. (a) HAMD scores in the study and control groups before and after therapy. (b) HAMA scores in the study and control groups before and after therapy. (c) PSQI scores in the study and control groups before and after therapy. ^*∗∗*^*p* < 0.01.

**Table 1:** Demographic characteristics of included participants.

Demographic characteristics	Study group (*n* = 47)	Control group (*n* = 44)	*p* value
	mean ± SD	mean ± SD	
Age (year)	49.47 ± 2.91	49.57 ± 2.93	0.87
Duration of perimenopausal state	2.49 ± 1.14	2.52 ± 1.17	0.90
BMI (kg/m^2^)	22.09 ± 1.70	21.86 ± 1.75	0.53
History of alcohol (Y/N)	6/42	4/40	0.74
History of smoking (Y/N)	3/44	4/41	0.71

**Table 2:** Uterine volume and endometrial thickness in the two groups before and after treatment.

	Study group (*n* = 47)	Control group (*n* = 44)	*p* value^a^
*Uterine volume (mm * ^*3*^ * )*			
Baseline	29.03 ± 4.98	29.43 ± 6.20	0.74
After treatment	29.78 ± 6.09	29.35 ± 6.90	0.76
*P* value^b^	0.23	0.89	

*Endometrial thickness (mm)*			
Baseline	2.41 ± 0.85	2.56 ± 0.73	0.40
After treatment	2.51 ± 0.81	2.53 ± 0.87	0.90
*P* value^b^	0.34	0.79	

^a^Independent *T*-test used; ^b^Paired Sample *T*-test applied.

**Table 3:** LH, FSH, E2, and melatonin levels before and after treatment in the two groups.

	Study group (*n* = 47)	Control group (*n* = 44)	*p* value^a^
*LH (mIU/mL)*			
Baseline	34.84 ± 11.93	36.52 ± 9.90	0.47
Post-therapy	21.01 ± 7.21	36.57 ± 12.38	<0.01^*∗∗*^
*P* value^b^	<0.01^*∗∗*^	0.95	

*FSH (mIU/mL)*			
Baseline	56.23 ± 11.89	58.08 ± 12.77	0.48
Post-therapy	36.27 ± 12.64	55.06 ± 12.93	<0.01^*∗∗*^
*P* value^b^	<0.01^*∗∗*^	0.10	

*E2 (pg/ml)*			
Baseline	43.75 ± 15.55	47.94 ± 16.33	0.21
Post-therapy	43.01 ± 13.48	46.97 ± 13.36	0.17
*P* value^b^	0.55	0.56	

*Melatonin (pg/ml)*			
Baseline	15.82 ± 3.32	15.79 ± 3.39	0.95
Post-therapy	16.03 ± 3.46	15.51 ± 3.20	0.46
*P* value^b^	0.77	0.71	

LH: luteinizing hormone, FSH: follicle generating hormone, E2: estradiol ^a^Independent *T*-test used ^b^Paired Sample *T*-test applied, ^*∗∗*^*p* < 0.01.

**Table 4:** Kupperman and MENQOL scores in the two groups before and after treatment.

	Study group (*n* = 47)	Control group (*n* = 44)	*p* value^a^
*Kupperman scores*			
Baseline	28.11 ± 4.45	27.39 ± 4.43	0.44
After treatment	12.68 ± 4.41	24.23 ± 4.97	<0.01^*∗∗*^
*P* value^b^	<0.01^*∗∗*^	<0.01^*∗∗*^	

*MENQOL scores*			
Baseline	54.30 ± 13.58	55.75 ± 15.27	0.63
After treatment	23.51 ± 8.29	50.52 ± 13.67	<0.01^*∗∗*^
*P* value^b^	<0.01^*∗∗*^	<0.01^*∗∗*^	

^a^Independent *T*-test used ^b^Paired Sample *T*-test applied, ^*∗∗*^*p* < 0.01.

**Table 5:** HAMD, HAMA, and PSQI scores in the two groups before and after therapy.

	Study group (*n* = 47)	Control group (*n* = 44)	*p* value^a^
*HAMD scores*			
Baseline	19.64 ± 6.78	19.09 ± 7.48	0.72
After treatment	11.00 ± 3.45	18.95 ± 6.29	<0.01^*∗∗*^
*P* value^b^	<0.01^*∗∗*^	0.84	

*HAMA scores*			
Baseline	16.47 ± 5.42	15.61 ± 5.43	0.46
After treatment	9.51 ± 3.36	15.23 ± 4.67	<0.01^*∗∗*^
*P* value^b^	<0.01^*∗∗*^	0.25	

*PSQI scores*			
Baseline	11.55 ± 4.26	11.27 ± 3.94	0.75
After treatment	5.98 ± 2.53	11.86 ± 3.43	<0.01^*∗∗*^
*P* value^b^	<0.01^*∗∗*^	0.30	

^a^Independent *T*-test used ^b^Paired Sample *T*-test applied ^*∗∗*^*p* < 0.01.

**Table 6:** Adverse reactions before and after treatment in the two groups.

	Study group (*n* = 47)	Control group (*n* = 44)	*p* value^a^
Breast pain	5/42	3/41	0.72
Rash	3/44	4/40	0.71
Nausea and vomiting	3/44	4/40	0.71

^a^Pearson chi-squared test used.

## Data Availability

The data collected for this study are available from the corresponding author.
